# Preoperative Nutritional Risk Assessment for Predicting Complications after Radical Cystectomy plus Urinary Diversion for Bladder Cancer

This article has been retracted.

**DOI:** 10.1155/2022/2901189

**Published:** 2022-08-16

**Authors:** Xing Wei, Jia Wang, Haitao Liu, Weizhe Fan, Gang Guo

**Affiliations:** ^1^Department of Urology, The 3rd Medical Center of Chinese People's Liberation Army General Hospital, Beijing 100039, China; ^2^Department of Urology Surgery, The First Affiliated Hospital of Air Force Military Medical University, Xi'an, Shaanxi 710032, China

## Abstract

**Objective:**

To investigate the predictive value of preoperative nutritional risk assessment on the occurrence of complications after radical cystectomy plus urinary diversion for bladder cancer.

**Methods:**

Retrospective analysis of 178 patients with bladder cancer between July 2010 and March 2022 who underwent elective radical cystectomy plus urinary diversion was conducted. The occurrence of complications within 90 days after surgery was counted for all patients, and the postoperative complication rates of patients with and without nutritional risk were compared and analyzed. Also, logistic regression analysis was used to assess the relative risk coefficients of NRS-2002 and the occurrence of postoperative complications.

**Results:**

Comparison of clinicopathological characteristics and surgical conditions between the two groups showed that the proportion of combined diabetes mellitus, operative time, and postoperative hospital stay were higher in the nutritional risk group (NRS ≥3 score) than in the no nutritional risk group (NRS <3 score), while the preoperative blood albumin (ALB) level was lower than that in the no nutritional risk group (NRS <3 score). The results of multifactorial risk regression analysis showed that low preoperative ALB level and high NRS score were independent risk factors for postoperative complications in bladder cancer (*P* < 0.05).

**Conclusion:**

The NRS-2002 nutritional risk score has good predictive value for the incidence of postoperative complications in patients with bladder cancer and provides a scientific basis for perioperative nutritional support.

## 1. Preface

Bladder cancer is the most common malignant tumor in urology, which is divided into two types, non-muscle layer invasive bladder cancer (NMIBC) and muscle layer invasive bladder cancer (MIBC) [1, 2]. Under normal circumstances, the clinical symptom of bladder cancer is mainly manifested as intermittent painless hematuria which occurs throughout the urination, while some patients take bladder irritation symptoms (i.e., frequency, urgency, painful urination, and so on) or pelvic pain as the main symptoms [3, 4]. Currently, radical cystectomy combined with urinary diversion has become the main surgical method for MIBC and recurrent high-risk NMIBC [5]. This technique can reduce the recurrence rate and mortality of bladder cancer after surgery and improve the survival rate. However, due to the complexity of the combined surgery, the long operation time, and the large trauma to the patient's body, the incidence of postoperative complications is at a high level, which is detrimental to the patient's postoperative recovery and adversely affects the surgical outcome. Therefore, finding reliable indicators to predict the incidence of postoperative complications in patients with bladder cancer has become one of the hot spots in clinical research [6].

The NRS-2002 nutritional risk scoring system is a simple and easy tool for nutritional risk screening, which was already recommended by ESPEN in 2002 as the tool of choice for nutritional risk screening in hospitalized patients, and has since been gradually promoted worldwide [7]. In 2006, the Chinese Society of Parenteral and Enteral Nutrition (CSPEN) recommended the “current recommendation of the NRS-2002 as a tool for assessing nutritional risk” as level A evidence [8]. There is existing evidence that complications may decrease nutritional status of patients [9]. But whether changes of NRS-2002 nutritional risk score are related to complications after bladder cancer surgery is still not scientifically reported. On this basis, this study analyzed the value of NRS-2002 nutritional risk scoring system in predicting the complications after bladder cancer surgery. The results are now reported as follows.

## 2. Information and Methods

### 2.1. Study Population and Grouping

The method of this study was retrospective case analysis, and we retrospectively searched electronic medical record database system, and the time interval of the search was set from July 2010 to March 2022. A total of 207 adult patients who underwent inpatient treatment in our urology department during this period were retrieved, and all of them were clinically diagnosed with bladder cancer and had detailed clinical and follow-up records. All patients were then screened according to predefined inclusion and exclusion criteria, and a total of 178 patients were eventually enrolled in this study.

#### 2.1.1. Inclusion Criteria

1. Adult patients with clinical and first confirmed diagnosis of bladder cancer.
2. Received surgical treatment for the first time.
3. Surgical treatment option chosen as radical total bladder dissection combined with urinary flow diversion.
4. Patients with preoperative perfection of relevant laboratory, imaging, pathology, and other tests.
5. At least 18 years old.

#### 2.1.2. Exclusion Criteria

1. Pediatric patients.
2. Those with relapsed bladder cancer.
3. Patients who had received adjuvant radiotherapy or bladder irrigation prior to surgery.
4. The first surgical treatment plan was partial cystectomy or radical cystectomy for bladder cancer.
5. Intraoperative conversion to open surgery for radical cystectomy plus urinary diversion.

### 2.2. Methodology

#### 2.2.1. Data Collection

Patient data were collected through the hospital information management system, which included (1) preoperative general information: patient gender, age, BMI, NRS-2002 score, presence of hypertension, diabetes mellitus (DM), coronary heart disease (CHD), preoperative serum albumin (ALB), and hemoglobin (HB); (2) surgery-related information: operation time, intraoperative bleeding, intraoperative blood transfusion, surgical procedure (transabdominal open and transabdominal laparoscopic), urethral diversion method (ileal neobladder (IN) and ileal cystectomy (IC)), tumor site, postoperative pathological staging; and (3) prognostic information: postoperative complications, hospitalization time, etc.

#### 2.2.2. Preoperative Nutritional Assessment

NRS-2002 was used for preoperative nutritional assessment, which included three aspects: disease severity score (0∼3), impaired nutritional status score (0∼3), and age score (0∼1). The final nutritional risk score was the sum of age score, impaired nutritional status score, and disease severity score. Those with a final score greater than or equal to 3 were considered to be at nutritional risk. Those with a final score less than 3 were considered to be patients without nutritional risk (the specific investigation methods are shown in Table 1).

#### 2.2.3. Definition of Postoperative Complications

The severity of postoperative complications was classified according to the Clavien–Dindo grading criteria: grade I did not require surgery, drugs, intervention, or endoscopy; grade II required drugs, blood transfusion, or total parenteral nutrition therapy; grade III required surgery, endoscopy, or intervention; grade IV could endanger the patient's life and required intensive care; and grade V led to the patient's death. Among them, grades I and II were defined as minor complications, and grades III to V were defined as serious complications [10].

### 2.3. Statistical Methods

SPSS 17.0 statistical software was used for data processing. Measurement data are expressed as mean ± standard deviation ($\bar{x}$ ± *s*), independent sample *t*-test is used for comparison between groups, count data are expressed as [*n* (%)], and chi-square (*χ*^2^) test is performed. Logistic regression analysis was used for multifactorial analysis of the risk of postoperative complications. The difference is statistically significant when *P* < 0.05.

## 3. Results

### 3.1. Comparison of Clinicopathological Characteristics

The 178 bladder cancer patients were grouped according to the NRS-2002 score, and those with NRS ≥3 were included in the nutritional risk group (62 patients, 34.83%), and those with NRS <3 were included in the no nutritional risk group (116 patients, 65.17%). There were no statistically significant differences in gender, age, BMI, presence of hypertension, coronary artery disease, ASA classification, preoperative hemoglobin, pathological grade, tumor size, and tumor location between the two groups (*P* > 0.05). The proportion of patients with combined diabetes mellitus and preoperative blood albumin levels were higher in patients with NRS ≥3 than in patients with NRS <3 (*P* < 0.05) (Table 2).

### 3.2. Comparison of Surgical Treatment

The operative times of patients in the nutritional risk group (NRS ≥3 points) and the patients in the no nutritional risk group (NRS <3 points) were (322.19 ± 46.04) min and (301.27 ± 40.12) min, respectively, and the postoperative hospital stays were (17.80 ± 4.90) d and (15.25 ± 4.02) d, respectively, and the differences between the two groups were statistically significant (*P* < 0.05). The differences in intraoperative bleeding, intraoperative blood transfusion, surgical procedure, urethral diversion method, and other surgical treatments between the two groups were not statistically significant (*P* > 0.05) (Table 3).

### 3.3. Comparison of Postoperative Complications

The complication rates in the NRS-2002 score ≥3 subgroup and the NRS-2002 score <3 subgroup were 54.84% (34/62) and 23.28% (27/116), respectively, and the differences were statistically significant (*P* < 0.05) when comparing the two groups (Table 4).

### 3.4. Analysis of Risk Factors for Postoperative Complications in Patients

The presence of postoperative complications in bladder cancer was used as the dependent variable, and five variables such as time to surgery, comorbid diabetes mellitus, preoperative blood albumin level, NRS score, and postoperative length of stay were used as independent variables in Tables 1–3 at *P* < 0.05 for regression analysis. The occurrence of postoperative complications was significantly correlated with patients' preoperative ALB levels (OR = 1.670, 95% CI: 1.331–2.097, *P* = 0.005) and NRS scores (OR = 2.787, 95% CI: 1.457–5.332, *P* < 0.001). Low preoperative ALB level and high NRS score were high risk factors for the development of postoperative complications in bladder cancer (Table 5).

## 4. Conclusion

As the most common malignant tumor in urinary system, bladder cancer patients with abnormal nutritional status are very common [11]. The reason is that with the proliferation of cancer cells, the body's nutritional consumption gradually increases. Moreover, after suffering from malignant tumor, the body has a series of stress reactions, which can cause metabolic abnormalities such as accelerated glucose utilization, insulin resistance, decreased muscle protein synthesis, and enhanced amino acid gluconeogenesis, thus aggravating nutritional abnormalities [12]. Radical cystectomy plus urinary diversion includes cystectomy, pelvic lymph node dissection, and urinary diversion, which is a complex procedure with a high incidence of postoperative complications that can seriously affect patients' physical recovery and even cause life-threatening conditions. In addition, patients at risk of abnormal nutritional status lack sufficient energy reserve, resulting in low immunity and poor anti-stress ability, so postoperative healing is slow and the incidence of complications is also increased [13]. A vicious circle can thus be formed between nutritional status and complications. So, preoperative assessment of patients' risk of postoperative complications and prognosis is particularly important [13].

More studies have pointed out age, BMI, duration of surgery, and urinary diversion method as risk factors associated with the occurrence of postoperative complications, and more factors are not modifiable and not very accurate [14, 15]. A study concluded that untimely albumin supplementation is a high risk factor for complications in patients in the perioperative period [16]. The results of our study showed that low preoperative serum albumin level is the high risk factor for postoperative complications of bladder cancer (*P* < 0.05). Serum albumin is one of the indicators of the nutritional status of the body, and its decrease can cause low immune function of the body, which can lead to symptoms such as delayed wound healing and infection [17]. This suggests that strict clinical monitoring of preoperative blood protein levels in patients with bladder cancer may help to reduce the incidence of postoperative complications.

Notably, the results of this study also showed that high NRS score was also a high risk factor for postoperative complications of bladder cancer (*P* < 0.05). This indicates that the nutritional status of the body is closely related to the incidence of postoperative complications in patients with malignant tumors [18, 19]. Further comparison of the severity of complications among patients with different NRS-2002 scores showed that the incidence of intestinal obstruction and the total incidence of complications in the NRS ≥3 group were significantly higher than those in the NRS <3 group (*P* < 0.05), with no significant differences in other groups.

NRS-2002 is the first nutritional risk screening tool developed on the basis of evidence-based medicine [20]. The scale was simple to operate and could be quickly evaluated in a short time through simple counseling. At the same time, the scale was less affected by subjective factors in the evaluation process, and the degree of acceptance by patients was high, so it had the advantage of high accuracy [21]. Karateke et al.'s study [22] demonstrated that the results of the clinical application of NRS-2002 were superior to other screening tools in terms of specificity and sensitivity. Raslan et al. [23] evaluated NRS-2002, MNA, and MUST nutritional screening in 705 patients and compared their ability to predict complications, mortality, and length of stay, respectively, and showed that NRS-2002 and MNA were superior to MUST in predicting clinical outcomes, while showing that NRS-2002 had better predictive power. This study further used logistic regression analysis to assess the relative risk coefficients of each clinical variable with the development of postoperative intestinal obstruction and found that low preoperative blood albumin levels and high NRS scores were high risk factors for the development of postoperative complications. This indicates that the NRS-2002 score has a good predictive value for complications after radical cystectomy combined with urethral diversion for bladder cancer.

In conclusion, the NRS-2002 nutritional risk score has good predictive value for the incidence of postoperative complications in bladder cancer patients and provides a scientific basis for perioperative nutritional support, which is recommended to be promoted. However, considering the relatively small sample included in this study, more randomized controlled studies with multiple samples are still needed to support the study, which is the direction of further research in this topic.

## Figures and Tables

**Table 1:** NRS scores.

Score	Nutritional status	Severity of disease	Age
0 points	Normal.	Normal.	＜70 years old
1 point	Weight loss of more than 5% in 3 months or eating 25% to 50% less than normal requirements in the previous week.	Fractures, chronic diseases such as liver cirrhosis, hemodialysis, general malignancies, diabetes, etc.	≥70 years old
2 points	Weight loss of more than 5% in 2 months or eating 50% to 75% less than normal requirements in the previous week.	Severe pneumonia, major abdominal surgery, shock, stroke, etc.	—
3 points	Weight loss of more than 5% in 1 month or more than 15% in 3 months or eating 75% to 100% less than normal requirement in the previous week or body mass index less than 18.50 Kg/m^2^.	Craniosynostosis, bone marrow transplantation, and ICU patients.	—

**Table 2:** Comparison of clinicopathological characteristics.

Information	NRS <3 (*n* = 116)	NRS≥3 (*n* = 62)	*t/χ * ^2^ value	*P* value
Age (years)	68.19 ± 9.44	66.40 ± 8.50	1.247	0.214

Gender (*n*, %)			1.367	0.242
Male	98 (84.48)	48 (77.42)		
Female	18 (15.52)	14 (25.81)		

BMI (kg/m^2^)	22.80 ± 5.42	21.79 ± 4.73	1.237	0.218

Hypertension (*n*, %)	43 (37.07)	16 (25.81)	2.313	0.128
DM (*n*, %)	7 (6.03)	10 (16.13)	4.766	0.029
CHD (*n*, %)	6 (51.72)	1 (1.61)	1.355	0.244

ASA grading (*n*, %)			0.517	0.772
Grade I	53 (45.69)	29 (46.77)		
Grade II	52 (44.83)	26 (41.94)		
Grade III∼IV	11 (9.48)	8 (12.90)		

Preoperative ALB (g/L)	42.23 ± 5.46	37.25 ± 4.03	6.318	0.000

Preoperative HB (g/L)	133.14 ± 12.30	130.58 ± 16.42	1.173	0.242

Pathological grade (*n*, %)			0.367	0.545
Low level	31 (26.72)	14 (22.58)		
High level	85 (73.28)	48 (77.42)		

Tumor size (cm)	4.70 ± 0.84	4.74 ± 0.63	0.329	0.743

Tumor site (*n*, %)			0.041	0.980
Side wall	89 (76.72)	46 (74.19)		
Triangle	20 (17.24)	11 (17.74)		
Bladder neck	7 (6.03)	4 (6.45)		

**Table 3:** Comparison of surgical treatment.

Information	NRS <3 (*n* = 116)	NRS≥3 (*n* = 62)	*t/χ * ^2^ value	*P* value
Operating time (min)	301.27 ± 40.12	322.19 ± 46.04	3.146	0.002
Intraoperative bleeding volume (mL)	397.59 ± 100.08	402.27 ± 103.30	0.294	0.769
Intraoperative blood transfusion (*n*, %)			0.258	0.612
Yes	26 (22.41)	16 (25.81)		
No	90 (77.59)	46 (74.19)		
Operation style (*n*, %)			0.854	0.356
Transabdominal open	10 (8.62)	3 (4.84)		
Transabdominal laparoscopic	106 (91.38)	59 (95.16)		
Urethral diversion method (*n*, %)			0.166	0.684
IN	34 (29.31)	20 (32.26)		
IC	82 (70.69)	42 (67.74)		
Postoperative hospital stay (*d*)	15.25 ± 4.02	17.80 ± 4.90	3.730	0.000

**Table 4:** Comparison of postoperative complications.

Information	NRS <3 (*n* = 116)	NRS≥3 (*n* = 62)	*χ * ^2^ value	*P* value
Grade I∼ II (*n*, %)				
Leaking of urine	2 (1.72)	3 (4.84)	1.436	0.231
Lung infection	2 (1.72)	2 (3.23)	0.415	0.520
Deep venous thrombosis	4 (3.45)	2 (3.23)	0.006	0.938
Electrolyte disturbance	5 (4.31)	3 (4.84)	0.026	0.871
Poor incision healing	3 (2.59)	3 (4.84)	0.629	0.428
Abdominal infection	2 (1.72)	2 (3.23)	0.415	0.520
Renal insufficiency	3 (2.59)	2 (3.23)	0.061	0.806

Grade III (*n*, %)				
Intestinal fistula	0 (0.00)	1 (1.61)	1.882	0.170
Intestinal obstruction	5 (4.31)	9 (14.52)	5.807	0.016

Grade IV (*n*, %)				
Infectious shock	1 (0.86)	1 (1.61)	0.205	0.651
Pulmonary embolism	0 (0.00)	2 (3.23)	3.785	0.052
Sepsis	0 (0.00)	1 (1.61)	1.882	0.170

Grade V (*n*, %)				
Postoperative death	0 (0.00)	1 (1.61)	1.882	0.170
Total complications (*n*, %)	27 (23.28)	34 (54.84)	17.869	0.000

**Table 5:** Analysis of risk factors for postoperative complications in patients.

Indicators	B	SE	Wald *χ*^2^	*P* value	OR	95% CI
Surgery time	0.245	0.182	1.258	0.230	1.278	0.894∼1.825
DM	0.013	0.007	3.231	0.070	1.013	0.997∼1.029
Preoperative ALB	0.513	0.116	8.136	0.005	1.670	1.331∼2.097
NRS score	1.025	0.331	15.587	＜0.001	2.787	1.457∼5.332
Postoperative hospital stay	0.412	0.383	2.240	0.110	1.510	0.713∼3.198

## Data Availability

The data can be obtained from the corresponding author upon reasonable request.
